The article "A PLA2R-IgG4 Antibody-Based Predictive Model for Assessing Risk Stratification of Idiopathic Membranous Nephropathy" was published in 2021. Journal: J Healthc Eng.

# A PLA2R-IgG4 Antibody-Based Predictive Model for Assessing Risk Stratification of Idiopathic Membranous Nephropathy

**DOI:** 10.1155/2021/1521013

**Published:** 2021-08-31

**Authors:** Xiaobin Liu, Jing Xue, Xiaoyi Guo, Yijie Ding, Yi Zhang, Xiran Zhang, Yiqing Huang, Biao Huang, Zhigang Hu, Guoyuan Lu, Liang Wang

**Affiliations:** ^1^Department of Nephrology, The First Affiliated Hospital of Soochow University, Suzhou 215006, China; ^2^Department of Nephrology, The Affiliated Wuxi People's Hospital of Nanjing Medical University, Wuxi 214023, China; ^3^Yangtze Delta Region Institute (Quzhou), University of Electronic Science and Technology of China, Quzhou 324000, China; ^4^NHC Key Laboratory of Nuclear Medicine, Jiangsu Key Laboratory of Molecular Nuclear Medicine, Jiangsu Institute of Nuclear Medicine, Wuxi 214063, China; ^5^College of Life Sciences and Medicine, Zhejiang Sci-Tech University, Hangzhou 310018, China; ^6^Medical Laboratory, The Affiliated Wuxi Children's Hospital of Nanjing Medical University, Wuxi 214023, China; ^7^Medical Laboratory, The Affiliated Wuxi People's Hospital of Nanjing Medical University, Wuxi 214023, China

## Abstract

**Background:**

Known as an autoimmune glomerular disease, idiopathic membranous nephropathy (IMN) is considered to be associated with phospholipase A2 receptor (PLA2R) in terms of the main pathogenesis. The quantitative detection of serum PLA2R-IgG and PLA2R-IgG4 antibodies by time-resolved fluoroimmunoassay (TRFIA) was determined, and the value of them, both in the clinical prediction of risk stratification in IMN, was observed in this study.

**Methods:**

95 patients with IMN proved by renal biopsy were enrolled, who had tested positive for serum PLA2R antibodies by ELISA, and the quantitative detection of serum PLA2R-IgG and PLA2R-IgG4 antibodies was achieved by TRFIA. All the patients were divided into low-, medium-, and high-risk groups, respectively, which were set as dependent variables, according to proteinuria and renal function. Random forest (RF) was used to estimate the value of serum PLA2R-IgG and PLA2R-IgG4 in predicting the risk stratification of progression in IMN.

**Results:**

Out-of-bag estimates of variable importance in RF were employed to evaluate the impact of each input variable on the final classification accuracy. The variable of albumin, PLA2R-IgG, and PLA2R-IgG4 had high values (>0.3) of 0.3156, 0.3981, and 0.7682, respectively, which meant that these three were more important for the risk stratification of progression in IMN. In order to further assess the contribution of PLA2R-IgG and PLA2R-IgG4 to the model, we built four different models and found that PLA2R-IgG4 played an important role in improving the predictive ability of the model.

**Conclusions:**

In this study, we established a random forest model to evaluate the value of serum PLA2R-IgG4 antibodies in predicting risk stratification of IMN. Compared with PLA2R-IgG, PLA2R-IgG4 is a more efficient biomarker in predicting the risk of progression in IMN.

## 1. Introduction

Idiopathic membranous nephropathy (IMN), known as primary membrane nephropathy, is the most common cause of primary nephropathy syndrome in adults [1, 2], which is approximately 20%∼30% of all the renal pathological biopsy reports [3]. IMN is usually manifested as nephropathy syndrome and depends on renal biopsy in diagnosis [4]. Although the study demonstrated that patients with IMN who received only symptomatic treatment had a relatively benign course, end-stage renal disease developed in 16% of the patients during a 5-year follow-up [5]. Therefore, it is critical to identify the degree of disease activity and progression risk in patients with IMN.

In 2009, Beck et al. [6] found 70% of the patients with IMN had antibodies against a conformation-dependent epitope in M-type phospholipase A2 receptor (PLA2R) which was present in normal podocytes and colocalized with IgG4 in immune deposits in glomeruli. Currently, PLA2R antibodies have been confirmed to be major pathogenic antibodies in IMN [7], which are mainly IgG4, and the titer levels of anti-PLA2R antibodies are related to the activity of the disease [8, 9]. In 2019, Kidney Disease Improving Global Outcomes (KDIGO) recommended that quantitative detection and regular follow-up of anti-PLA2R antibodies would contribute to differential diagnosis and assessment of activity in IMN [10].

At present, the detection of sera anti-PLA2R antibodies normally applies indirect immunofluorescence assay (IIFA) and enzyme-linked immunosorbent assay (ELISA) [11]. IIFA is not a quantitative detection measure, while ELISA is characterized by low detection sensitivity [12]. In 2017, Huang et al. [13] developed an ultrasensitive quantitative assay, using time-resolved fluoroimmunoassay (TRFIA), for the detection of anti-PLA2R-IgG testing. Establishing the cutoff value for anti-PLA2R-IgG of 1990 ng/mL, the diagnostic sensitivity and specificity in IMN were 74% and 100%, respectively. Huang et al. [14] further tested anti-PLA2R-IgG4 and found that the diagnostic sensitivity and specificity in IMN were 90% and 100%, respectively when established the cutoff value for anti-PLA2R-IgG4 of 161.2 ng/mL.

In this study, we determined the quantitative detection of anti-PLA2R-IgG and -IgG4 antibodies by TRFIA and observed the value of them both in the clinical prediction of different risk-stratified IMN.

## 2. Materials and Methods

### 2.1. Subjects Selection

A total of 95 patients with IMN proved by renal biopsy, who had tested positive for serum PLA2R antibodies by ELISA, from the Affiliated Wuxi People's Hospital of Nanjing Medical University, were enrolled from January 2016 to December 2017. According to proteinuria <4 g/d, 4–8 g/d, and >8 g/d, with renal function taken into consideration, all the patients were divided into low-, medium-, and high-risk groups, respectively [15].

Blood samples were collected before renal biopsy and before the immunosuppressive therapy, which were left standing to clot thoroughly before centrifuging at 3000 rpm/min for 4 min to obtain serum, and sera were then stored at −80°C for pending analysis. All renal tissue specimens were examined using light microscope, immunofluorescence, and electron microscope. Pathological grading was performed by Ehrenreich and Churg standards [16].

Goat anti-human IgG antibodies were obtained from Jackson ImmunoResearch (USA), and mouse anti-human IgG4 antibodies were offered by Hytest (Finland). Europium labeling kits (1244-302) were purchased from Perkin Elmer (USA). The polystyrene microtiter plates were obtained from Nunc International (Denmark). The recombinant PLA2R antigen, series of standards of anti-human PLA2R-IgG and PLA2R-IgG4 were prepared in our laboratory as previously reported [13, 14]. All the buffer solutions were supplied from Jiangyuan Co. (China). The other reagents were of analytical grade and obtained from Sinopharm Chemical Reagent (China). An AutoDELFIA_1235_ was purchased from Perkin Elmer (USA).

### 2.2. Anti-PLA2R-IgG and PLA2R-IgG4 Detection Procedure

Firstly, 100 *μ*L of standards or diluted sera were pipetted to the microtiter plates fixed with 5 *μ*g/mL of rPLA2R. The working dilutions of serum samples were 1 : 200 and 1 : 20 in the anti-PLA2R-IgG and anti-PLA2R -IgG4 assays, respectively. The mixture was reacted with continuously shaking at 25°C for 1 h. After the unreacted substances were removed by washing for 3 times, the plates were pipetted with europium-labelled goat anti-human IgG or mouse anti-human IgG4 antibodies, shaken for 1 h at 25°C, and then rinsed for 6 times. Finally, 96-well plates were added with 200 *μ*L of enhancement solution, agitated for 5 min, and measured in AutoDELFIA_1235_. The concentrations of serum samples of anti-PLA2R-IgG and anti-PLA2R-IgG4 were automatically calculated from the fluorescence of wells by AutoDELFIA_1235_. According to the previous work [13, 14], the cutoff values were 1990 ng/mL and 161.2 ng/mL for anti-PLA2R-IgG and anti-PLA2R-IgG4, respectively.

### 2.3. Statistical Analyses

This work employed 38 features (variables) including pathological and clinical features to describe the patients' characters, which contained mean, standard deviation, and correlation coefficient of samples as shown in Table 1. The three groups (low-, medium-, and high-risk groups), which were divided according to proteinuria and renal function, were set as dependent variables. The results demonstrated that PLA2R-IgG (0.394) and PLA2R-IgG4 (0.524) had great correlation coefficients with the dependent variables. In our study, the number of patients in class 1, 2, and 3 (three types of risk stratification) was 45, 41, and 9, respectively.

### 2.4. Random Forest

In machine learning, the random forest (RF) [17] is a classifier that contains multiple decision trees, and the output category is determined by the mode of the category output by the individual trees. In this work, random forest was used as an analysis and classification tool to estimate the value of serum PLA2R-IgG and PLA2R-IgG4 in predicting the risk stratification of progression in IMN. Compared with *k*-nearest neighbor (KNN) and support vector machines (SVM) classifiers, it has the following advantages: (1) it can assess the importance of variables when determining categories; (2) when building a forest, it can produce an unbiased estimate of the generalized error internally; (3) for unbalanced classification data sets, it can balance errors; (4) the learning process is fast.

## 3. Results

### 3.1. Evaluation Measurements

The accuracy (ACC) is utilized to evaluate the performance of the RF model under 5-fold cross-validation (5-CV). The calculation method of ACC is as follows:

(1) $$\begin{array}{c} \text{whole ACC}=\frac{\sum_{i=1}^{c}TP^{i}}{M}\times 100\%,\\ {\text{ACC}}^{i}=\frac{TP^{i}}{M^{i}}\times 100\%,\\ M=\sum_{i=1}^{c}M^{i}, \end{array}$$

where *c* denotes the number of classes. *TP*^*i*^ denotes the number of true positive (TP) in subclass *i*. *M* and *M*^*i*^ denote the number of whole test samples and subclass test samples. ACC^*i*^ denotes the accuracy in subclass *i*.

### 3.2. Relative Importance of Inputs in Estimating IMN

To evaluate the impact of each input variable on the final classification accuracy. We employed out-of-bag estimates of variable importance in RF. The RF stored the increase in mean square error (MSE) averaged over all trees in the ensemble and divided by the standard deviation taken over the trees, for each variable. So, we could get the importance scores of all input variables. In general, the larger the score, the more important it is for the prediction model.  Figure 1 shows the results of relative importance for inputs. It could be seen from the figure that the 21-th (albumin), 37-th (PLA2R-IgG), and 38-th (PLA2R-IgG4) variables had high values (>0.3) of 0.3156, 0.3981, and 0.7682, respectively.

### 3.3. Comparison of PLA2R-IgG and PLA2R-IgG4

In order to further evaluate the contribution of PLA2R-IgG and PLA2R-IgG4 to the model, we constructed four different models, which contain both PLA2R-IgG and PLA2R-IgG4 variables, PLA2R-IgG variable, PLA2R-IgG4 variable, and no PLA2R- IgG and PLA2R-IgG4 variables. The relevant information of the models is shown in Table 2.

The classification performance of the 4 models was verified by 5-fold cross-validation. And, the results are listed in Table 3. Obviously, when PLA2R-IgG and PLA2R-IgG4 were included, the prediction performance of the model (model 1) was the best, and the overall classification accuracy was 0.6743. In the overall ACC, the performance of model 2 (0.6422) was not better than model 3 (0.6639). This further verified that PLA2R-IgG4 is more important than PLA2R-IgG for classification accuracy. In addition, the performance of the model (model 4) was the worst (0.6290), when PLA2R-IgG4 and PLA2R-IgG were not contained at the same time. From the above test, it could be found that PLA2R-IgG and PLA2R-IgG4 were very helpful for classification. However, PLA2R-IgG4 could achieve better results than PLA2R-IgG.

In this study, we employed *t*-test to evaluate the significant differences of average ACC between different models. The results were list in Table 4, which show that the differences between model 1 and other three models were significant. Furthermore, the *P* value of model 3 and model 4 was 0.0022. This means that the PLA2R-IgG4 feature had a more significant performance improvement compared to the ordinary model (without PLA2R-IgG and PLA2R-IgG4).

## 4. Discussion

It is widely recognized that IMN is an autoimmune glomerular disease in which autoantibodies combine with antigens on glomerular podocytes and deposit in glomerular capillary walls [18]. With the discovery of M-type phospholipase A2 receptor (PLA2R) which was identified as the major target antigen, progress was made in understanding the pathogenesis of IMN [6]. Circulating anti-PLA2R antibodies not only contribute to distinguish primary membranous nephropathy from secondary membranous nephropathy in diagnosis but also conduce to monitor the immunological activity degree during the treatment period [19]. Accordingly, the quantitative detection of circulating anti-PLA2R antibodies is particularly important in diagnosis and treatment of IMN.

Among all the PLA2R-IgG antibodies, PLA2R-IgG4 antibodies are predominant [6, 18]. Lacking of mature commercial testing means TRFIA was employed in this study for the quantitative detection of anti-PLA2R-IgG4 antibodies. As a novel nonisotopic labeling technology, TRFIA has the advantages of high sensitivity (10^−18^ mol/L), wide monitoring range, and less susceptibility to matrix interference [14]. Our previous work discovered that using the cutoff value of 161.2 ng/mL, anti-PLA2R-IgG4 had higher sensitivity in diagnosis than anti-PLA2R-IgG by the cutoff value of 1990 ng/mL (90% versus 74%) [14]. Therefore, we speculate that, in addition to anti-PLA2R-IgG, anti-PLA2R-IgG4 may be an efficient biomarker in the assessment of the severity and prognosis of IMN too.

In recent years, machine learning methods have been widely used in medicine [20–22] and biology [23–25] to solve difficult data analysis problems for researchers. In our study, RF was employed to evaluate the importance of all the features (input variables). And, we found that the 21th (albumin), 37th (PLA2R-IgG), and 38th (PLA2R-IgG4) variables had high values (>0.3) of 0.3156, 0.3981, and 0.7682, respectively, which meant these three features were more important to the risk stratification of progression in IMN. At the same time, as shown in Figure 1, PLA2R-IgG4 manifested a better predictive value compared with PLA2R-IgG (0.7682 versus 0.3981). In addition, it could be seen from Table 3 that the prediction effect of the PLA2R-IgG4 feature (0.6639) was better than that of the PLA2R-IgG feature (0.6422). When both PLA2R-IgG4 and PLA2R-IgG features were input into the model, its prediction performance was the best (0.6743). The above test results further validated the importance of PLA2R-IgG4 and PLA2R-IgG in assessing the risk level model. In Table 4, we evaluated the significant differences between different models. Obviously, the difference between model 1 and other models was significant (*P* value < 0.05). Compared with model 4, model 3 also had significant difference (*P* value = 0.0022). It was obvious that PLA2R-IgG4 played an important role in improving the predictive ability of the model.

## 5. Conclusions

In this study, we evaluated the value of serum PLA2R-IgG4 antibodies in predicting risk stratification of IMN by establishing a random forest model. Compared with PLA2R-IgG, PLA2R-IgG4 is a more efficient biomarker in predicting the risk of progression in IMN. The study results are satisfactory, while disadvantages remain (1) there is lack of analysis about the value of serum PLA2R-IgG4 in the prediction of treatment effect; (2) the sample size needs to be further expanded to minimize the prediction bias. In the next work, we will expand the sample size and survey the predictive effect of serum PLA2R-IgG4 in the therapeutic regimen and prognosis of IMN.

## Figures and Tables

**Figure 1:** Relative importance for inputs.

**Table 1:** The information of data set.

No.	Feature (variable)	Value	*r* ^*∗*^
1	Age (years)	55.110 ± 15.110	0.175
2	Gender (males/females)	56/39	0.105
3	Renal tubular atrophy score	1.057 ± 0.721	0.080
4	Renal interstitial fibrosis score	1.100 ± 0.731	0.113
5	Renal interstitial lymphoplasmacytic infiltrate score	1.068 ± 0.861	0.187
6	Total score of renal tubular and interstitium	3.236 ± 2.138	0.136
7	Pathological stage of IMN	1.452 ± 0.495	0.009
8	IF IgA	0.220 ± 0.477	0.089
9	IF IgM	0.252 ± 0.635	0.034
10	IF IgG	2.789 ± 0.697	0.009
11	IF C1q	0.242 ± 0.488	0.098
12	IF C3	1.205 ± 0.738	−0.035
13	Renal tissue PLA2R antigen	0.952 ± 0.357	−0.031
14	SBP (mmHg)	133.389 ± 14.973	0.017
15	DBP (mmHg)	79.989 ± 9.079	−0.109
16	Serum C3 (mg/L)	894.305 ± 253.312	−0.008
17	Serum C4 (mg/L)	241.147 ± 87.192	0.058
18	Serum IgA (g/L)	5.206 ± 28.002	0.061
19	Serum IgG (g/L)	7.084 ± 2.891	−0.077
20	Serum IgM (g/L)	1.257 ± 0.637	−0.013
21	Serum albumin (g/L)	23.335 ± 8.233	−0.449
22	Hematuria (/uL)	102.377 ± 138.301	−0.014
23	Serum creatinine (umol/L)	83.664 ± 34.042	0.168
24	eGFR-EPI (ml/min)	86.535 ± 24.060	−0.189
25	BUN (mmol/L)	4.986 ± 1.929	0.172
26	Serum glucose (mmol/L)	5.142 ± 0.810	0.321
27	Serum lithic acid (umol/L)	344.676 ± 89.678	0.048
28	TG (mmol/L)	2.406 ± 1.471	0.415
29	TC (mmol/L)	7.119 ± 2.289	0.141
30	LDL-C (mmol/L)	3.902 ± 1.379	0.077
31	HDL-C (mmol/L)	1.323 ± 0.432	−0.110
32	WBC (×10^9^/L)	8.577 ± 13.978	0.088
33	Hemoglobin (g/L)	122.204 ± 24.962	0.058
34	PLT (×10^9^/L)	219 ± 65.409	−0.104
35	C-reactive protein (mg/L)	2.807 ± 3.167	0.057
36	ESR (mm/H)	53.589 ± 34.176	0.233
37	Serum PLA2R-IgG (ng/mL)	5243.957 ± 9282.902	0.394
38	Serum PLA2R-IgG4 (ng/mL)	1762.615 ± 2662.328	0.524

^*∗*^denotes that each feature correlated with risk stratification of progression in IMN using Pearson correlation coefficient (*r*).

**Table 2:** The information of models.

Model	Number of features (variables)	
Model 1	38	With PLA2R-IgG and PLA2R-IgG4
Model 2	37	With PLA2R-IgG and without PLA2R-IgG4
Model 3	37	Without PLA2R-IgG and with PLA2R-IgG4
Model 4	36	Without PLA2R-IgG and PLA2R-IgG4

**Table 3:** Comparison on four models via 5-fold cross-validation.

Model	Overall ACC	ACC^1^	ACC^2^	ACC^3^
Model 1	0.6743	0.8	0.6583	0.1
Model 2	0.6422	0.7778	0.5833	0.2
Model 3	0.6639	0.7778	0.6806	0
Model 4	0.6290	0.7556	0.6306	0

ACC^1^: the accuracy of class 1; ACC^2^: the accuracy of class 2; ACC^3^: the accuracy of class 3.

**Table 4:** Analysis of statistical significance for different methods via 5-fold cross validation (10 times).

	*P* value
Between model 1 and model 2	6.355*e* − 4
Between model 1 and model 3	0.0085
Between model 1 and model 4	1.8*e* − 5
Between model 2 and model 3	0.1142
Between model 2 and model 4	0.1510
Between model 3 and model 4	0.0022

## Data Availability

The data used to support the research can be obtained from the corresponding authors according to the requirements of the institution.
